The article "Exploring the Correlation between Changes in Gut Microbial Community Diversity and Depression in Human Populations" was published in 2022. Journal: Biomed Res Int.

# Exploring the Correlation between Changes in Gut Microbial Community Diversity and Depression in Human Populations

**DOI:** 10.1155/2022/6334868

**Published:** 2022-07-29

**Authors:** Xin Li, Ke Jing, Hong Lu, Ke Li, Yaowu Zhang, Hasichaolu

**Affiliations:** Department of Laboratory Medicine, The First Hospital of Shanxi Medical University, Taiyuan, China

## Abstract

Depression, also known as depressive disorder, is a group of psychosomatic affective disorders characterized by persistent and significantly depressed mood, delayed thinking, and cognitive impairment. The aim of this study was to explore the correlation between changes in gut microbial community diversity and depression to provide data on new strategies for the prevention and treatment of depression. In this study, we separated participants into a group of depressed patients and a healthy comparison group. We analyzed the gut microbial community structure of depressed patients and healthy comparisons using second-generation sequencing of the bacterial 16S RNA gene. There were significant differences in the gut microflora structure between patients with depression and healthy individuals. The gut flora alpha diversity index was significantly reduced in patients with depression compared to that in the healthy population. At the species level, the relative abundance of *Coprococcus catus* and *Bacteroides barnesiae* was significantly lower in the depressed group than that in the control group. The development of depression may be associated with a decrease in beneficial gut bacteria.

## 1. Introduction

Depression, also known as depressive disorder, is a group of psychosomatic affective disorders characterized by persistent and significantly depressed mood, delayed thinking, cognitive impairment, reduced volitional activity, and somatic symptoms [1]. The pathogenesis of depression remains unclear and is thought to be related to genetic, biochemical, neuroendocrine, immune, and environmental factors [2]. Some hypotheses of depression have gradually received increasing attention because the proposed biomarkers for depression may affect pharmacological treatments. These hypotheses include biomarkers implicated in the stress-responsive hypothalamic pituitary adrenal (HPA) axis, neuroendocrine systems, the neurotrophic family of growth factors, and neuroinflammation [3]. Mounting evidence has shown that stress-induced abnormalities of the HPA axis are associated with depression and cognitive impairment, owing to the increased secretion of cortisol and insufficient inhibition of glucocorticoid receptor regulatory feedback [4, 5]. Accumulating evidence suggests that the glutamate system is associated with the incidence of depression. Early studies have shown increased levels of glutamate in the peripheral blood, cerebrospinal fluid, and brain of depressed patients [6, 7], as well as N-methyl-D-aspartate receptor (NMDAR) subunit disturbances in the brain [8, 9]. A number of studies have shown that patients with depression have neurotransmission or functional defects in gamma-aminobutyric acid (GABA) [10, 11]. Many studies have shown that the microbiota-gut-brain axis (MGBA) plays an important role in regulating mood, behavior, and neuronal transmission in the brain [12, 13]. It has been reported that gut microbiome alterations are associated with depressive-like behaviors [14, 15] and brain function [16].

A large number of studies in recent years have found that the balance of the type, composition, and quantity of the gut microbial community are closely related not only to the health of the host but also to their behavior, and that dysbiosis of the gut flora may induce depression, anxiety, and cognitive disorders, including schizophrenia, Alzheimer's disease, and autism spectrum disorder [17–19]. Recent approaches in depression and anxiety research have investigated the influence of the gut microbiota on neurobiology and behavior. Research into the MGBA began with the observation that there is a high comorbidity of anxiety and depression in patients with inflammatory bowel disease [20, 21] and irritable bowel syndrome [22, 23]. In addition, gut microbiota composition in individuals with anxiety or depression has been shown to differ from that in healthy comparisons [24, 25], and animal models of depression show altered gut microbiota when compared with that of nondepressed controls [26].

In this study, we attempted to investigate the structure of the gut microbial community in depressed patients using molecular biology methods to preliminarily explore the correlation between gut microbial imbalance and the development of depression, provide valuable data on gut microecological regulation, and ultimately guide the efforts to prevent and treat clinical depression.

## 2. Materials and Methods

### 2.1. Participants

Seventy depressed patients who attended the First Hospital of Shanxi Medical University from December 2021 to January 2022 were selected as the depression group. According to medical history, clinical manifestations, and laboratory tests, the following diagnostic criteria were used: (1) diagnostic criteria in the International Statistical Classification of Diseases and Related Health Problems 10th Revision (ICD-10) [27] were met; (2) symptoms were mainly depressed mood with at least four of the following: unpleasant feelings or loss of interest; fatigue or loss of energy; psychomotor retardation or agitation; feelings of guilt, self-blame, or low self-esteem; reduced ability to think or difficulty with cognitive association; self-injury, suicidal behavior, or recurrent thoughts of death; sleep disorders, such as early awakening, insomnia, or excessive sleep; decreased libido; decreased sexual desire; decreased sleepiness; and significant weight loss or decreased appetite; and (3) a Hamilton Depression Scale score ≥ 20. Inclusion criteria were meeting the above diagnostic criteria as confirmed by our specialist, duration of illness ≥ 2 weeks, and age ≥ 18 years. Exclusion criteria were underlying diseases such as hypertension, coronary heart disease, metabolic diseases, liver cirrhosis, inflammatory bowel disease, irritable bowel syndrome, and other psychiatric diseases, such as bipolar disorder, persistent mood disorder, and manic episodes. All enrolled subjects avoided antidiarrheal drugs, bloating agents, probiotics, antispasmodics, antibiotics, and other medications within 30 days prior to sample collection.

Twenty-two healthy individuals who underwent health checkups at the First Hospital of Shanxi Medical University from December 2021 to January 2022 were selected as healthy comparisons. The inclusion criteria were no chronic diarrhea, no special dietary preferences, and no underlying diseases, such as hypertension, diabetes mellitus, and hyperlipidemia. Exclusion criteria were abnormal mental status, menopausal syndrome, neurosis, long-term insomnia, or antibiotic treatment within two weeks before the physical examination.

Both groups of study subjects voluntarily enrolled in this study, and an informed consent agreement was executed with every participant. The subject recruitment process is illustrated in Figure 1. There was no statistical difference between the two groups in terms of general information (*p* > .05). This study was reviewed and approved by the Medical Ethics Committee of the First Hospital of Shanxi Medical University.

### 2.2. Stool Collection and DNA Extraction

Stool sample collection was completed within 24 hours of admission for the inpatients in the depression group. Stool (approximately 15 g) was collected in a sterile plastic box, numbered, registered, and stored in a refrigerator at -80°C. In the healthy comparison group, the samples were collected and processed similarly upon completion of a physical examination. After all stool specimens were collected, DNA was extracted using a stool DNA extraction kit (StoolGen DNA kit, Beijing Youji Technology Co., Ltd.). The extracted total DNA was tested for integrity using an agarose gel electrophoresis instrument (Beijing Liuyi Company, DYY-6C).

### 2.3. DNA Amplification

We amplified different regions of the bacterial 16S rDNA gene and other functional genes using polymerase chain reaction (PCR). Primers were designed to amplify single or multiple variable regions of the rRNA gene using conserved regions of ribosomal RNA to sequence and analyze microbial diversity. In this experiment, the highly variable V3-V4 region of the bacterial 16S rRNA gene, with a length of approximately 468 bp, was used for sequencing. PCR amplification was performed using bacterial 16S rDNA V3-V4 region-specific primers 338F (5′-ACTCCTACGGGAGGCAGCA-3′) and 806R (5′-GGACTACHVGGGTWTCTAAT-3′). The barcode in the preprimer is a 7-base oligonucleotide sequence used to distinguish different samples from the same library. PCR amplification was performed using the Q5 DNA high fidelity polymerase (NEB, M0491L), and the amplification reaction system is shown in Table 1.

After the required components of the PCR reaction were configured, the template DNA was predenatured at 98°C for 30 seconds on the PCR instrument in order to denature the template DNA to a sufficient degree prior to entering the amplification cycle. In each cycle, the sample was held at 98°C for 15 seconds to denature the template, then the temperature was lowered to 50°C and held for 30 seconds to fully anneal the primers to the template. Then, the sample was held at 72°C for 30 seconds to extend the primers over the template and synthesize the DNA. This method makes up a single PCR cycle. The cycle was repeated 25-27 times to allow a large accumulation of amplified DNA fragments. Finally, the product was kept at 72°C for 5 minutes to allow complete extension and was stored at 4°C. The amplification results were subjected to 2% agarose gel electrophoresis, and the target fragments were cut and recovered using the Axygen gel recovery kit.

### 2.4. PCR Product Quantification and Mixing

The PCR products were quantified on a microplate reader (BioTek, FLx800T) using the Quant-iT PicoGreen dsDNA Assay Kit (Invitrogen, p7589) and then mixed according to the amount of data required for each sample.

### 2.5. Library Construction

1. Library construction was performed using the TruSeq Nano DNA LT Library Prep Kit (Illumina). End repair was first performed using the End Repair Mix2 feature of the kit to excise the base protruding from the 5′ end of the DNA and fill in the missing base at the 3′ end, while adding a phosphate group at the 5′ end. The method involved the following three steps in sequence: (a) the mixed DNA fragments (30 ng) were rehydrated to 60 *μ*L and 40 *μ*L with the End Repair Mix2 feature; (b) DNA fragments were mixed with microsampler blast and incubated on a PCR instrument at 30°C for 30 minutes; and (c) the end-repair system was purified using BECKMAN AMPure XP beads and eluted with 17.5 *μ*L of a resuspension buffer
2. Adenine bases (A) were added at the 3′ end of the DNA sequences to prevent self-connection of the DNA fragments and ensure that the DNA would connect to a sequencing junction with a prominent thymine base (T) at the 3′ end using the following method: (a) 12.5 *μ*L of A-tailing mix was added to the fragment-selected DNA; (b) the samples were mixed well with a microsampler blow, placed on a PCR instrument, and incubated with the following temperature schedule: 37°C for 30 minutes, 70°C for 5 minutes, 4°C for 5 minutes, and 4°C indefinitely
3. A splicing agent with a specific label was added. This procedure was performed to allow final hybridization of the DNA to the flow cell as follows: (a) 2.5 *μ*L of a resuspension buffer, 2.5 *μ*L of a ligation mix, and 2.5 *μ*L of a DNA adapter index were added to the system to which A had been added; (b) the solution was mixed with a microsampler blow and incubated at 30°C for 10 minutes on a PCR instrument; (c) 5 *μ*L of stop ligation buffer was added to the mixture; and (d) the system with added connectors using BECKMAN AMPure XP beads was purified
4. The DNA fragment that had been coupled by PCR was amplified, and the PCR system was purified using BECKMAN AMPure XPbeads
5. Final fragments were selected, and the library was purified using 2% agarose gel electrophoresis

### 2.6. Library Quality Control and Sequencing

1. Library quality control (QC) and quantification were performed using the following method: a 1 *μ*L sample of the library was taken, and the library was subjected to 2100 QC using the Agilent High Sensitivity DNA Kit on an Agilent Bioanalyzer (Agilent Technologies, USA) machine, wherein qualified libraries were expected to have a single peak and no junction. The libraries were quantified using the Quant-iT PicoGreen dsDNA Assay Kit on a QuantiFluor fluorometer (Promega), wherefrom qualified libraries demonstrated a calculated concentration of 2 nM or more
2. The library was sequenced using the following method: for qualified libraries, 2 × 250 bp double-end sequencing was performed on a MiSeq machine using the MiSeq Reagent Kit V3 (600 cycles). Libraries on the machine (Index not reproducible) were gradient diluted to 2 nM and mixed in proportion to the amount of data required. The mixed libraries were denatured to single strands using 0.1 N NaOH for upsequencing. The amount of uploaded library was controlled to be between 15 and 18 pM. The data obtained from the down machine were subjected to bioinformatics analysis

### 2.7. Bioinformatics Analysis

The off-board data were filtered, and the original sequencing data were processed using an internally written program to filter out low-quality sequencing fragments (reads). The remaining high-quality clean data were used for postanalysis with the following steps:

1. 30 bp was set as the window length. If the window began truncating read end sequences, we removed the final read length below 75% of the reads
2. The Fast Length Adjustment of Short reads (FLASH) (v1.2.11) software was used to overlap the DNA fragments and assemble pairs of reads obtained from the double-end sequencing into a single sequence, resulting in high complexity reads
3. After obtaining the operational taxonomic unit (OTU) representative sequences, the OTU representative sequences were compared with the Greengene_2013_5_99 database using RDP Classifier (v2.2) software
4. The OTUs were annotated with their respective species and compared

### 2.8. Analysis of Microbial Community Diversity and Abundance in the Gut

The generated OTU information was used to analyze the community diversity and abundance variation of the gut microflora. Alpha diversity values of the samples were calculated using Mothur (v1.31.2) software, including the observed species index, Chao index, ACE index, Shannon index, and Simpson index, where the observed species index, Chao index, and ACE index reflected the abundance of the community in the samples. The Shannon index and the Simpson index reflected the diversity of the community. In addition, the relative abundance of each OTU in each sample was calculated based on their abundance. This abundance information was used to carry out a principal component analysis (PCA) of the OTUs by analyzing the composition of the different sample OTUs (97% similarity) to reflect the differences and distances of samples. PCA uses variance decomposition to reflect the differences of multiple sets of data on a two-dimensional coordinate graph. The axes reflect the maximum variance value of two eigenvalues; if two samples are closer on the graph, it means that the composition of these two samples are more similar.

Species classification of the OTUs was performed, and heat map clustering analysis was performed at several taxonomic levels of phylum, order, family, genus, and species, respectively, by comparison with the database. Differences in microbial community abundance between samples from the depression and healthy comparison groups were examined statistically, and the significance of the differences was assessed using the false discovery rate (FDR), from which the species responsible for the differences in the composition of the two groups could be screened. We used R software (rank sum test, Fisher's exact test, *t*-test, and variance test) for the analysis of significant differences between the groups, and *p* value correction was performed by *p*.adjust in the R (v3.1.1) package, using the Benjamini-Hochberg (BH) correction method.

## 3. Results

### 3.1. General Information on the Subjects Included in the Study

The characteristics of the subjects included in this study are shown in Table 2. Forty patients with depression and 22 healthy individuals were included in this study. There were 15 males and 25 females in the depression group, aged 18 to 65 years, with a mean age of 37.9 ± 14.3 years. The healthy comparison group had 13 males and 9 females, aged 21 to 65 years, with a mean age of 44.0 ± 14.3 years. The mean age of the depression group was lower than that of the healthy comparison group. Blood test results showed no significant difference in total cholesterol, triglyceride, glucose, aspartate aminotransferase, and alanine aminotransferase levels between the two groups.

### 3.2. Sequence Length Distribution

16S rDNA sequencing of gut bacteria from the depression and healthy control samples yielded a total of 471,541 tags for all samples, with an average of 76,049 ± 5,419 tags per sample. The average tag length was 450 ± 8 bp. A total of 45,71642 tags remained for all samples, with an average of 73,736 ± 5,336 tags and an average length of 410 ± 8 bp.

### 3.3. OTU Number Statistics and Abundance Analysis

Clean tags processed as described above were clustered by OTU, and OTU species classification was completed by annotating the OTUs. Information on the abundance of each sample in each OTU was counted, and the abundance of the OTUs initially indicated the species richness of the samples (Table 3). Sixty-two samples from the depression and healthy comparison groups yielded a total of 1,404 OTUs, and an analysis of the OTU Venn diagrams yielded 356 OTUs in the depression group and 248 OTUs in the healthy comparison group, for a total of 800 OTUs in both groups (Figure 2).

The relative abundance of each OTU in each sample was calculated based on the abundance file of each OTU in each sample. This abundance information was used to perform a PCA of the OTUs, as can be seen in Figure 3. The first two principal components of this analysis explained 22.44% and 12.08% of the total variance, respectively. From this figure, it can be seen that the microbial community samples of the depression group and the healthy comparison group could not be clearly separated in the individual samples based on OTU.

### 3.4. Species Annotation Analysis

OTU species classification was carried out by comparison with the database and the area and histogram of species profiling for each sample at several taxonomic levels of phylum, order, family, genus, and species, respectively.  Figure 4 shows the species profiling of each sample at the different taxonomic levels. The proportion of different species in each sample can be visualized from the figure.

### 3.5. Sample Diversity Analysis between Groups

The Shannon and Simpson indices were used to analyze the diversity of the flora in the samples of the two groups. The diversity indices of the groups are presented in Table 4. From the Shannon index dilution curves and the Simpson index dilution curves of the two sequenced groups (Figure 5), it can be seen that the curves of all samples increased rapidly with the increase in the number of sequencing and eventually leveled off, indicating that the amount of sequenced data was large enough to reflect the majority of microbial information in the samples. The greater the Shannon index, the higher the diversity of the community in the samples. The Shannon index of the depression group was found to be significantly lower than that of the healthy comparison group (2.219 vs. 2.736, *p* < .05), as shown in Figure 6(a), indicating that the diversity of the community in the depression group was lower. The lower the value of the Simpson index, the higher the diversity in the samples. The Simpson index of the depression group colonies was found to be significantly greater than that of the healthy comparison group (0.267 vs. 0.169, *p* < .05), as shown in Figure 6(b), indicating a lower diversity of the depression group colonies, in agreement with the Shannon index findings.

Both the ACE and Chao indices were used to estimate the number of OTUs contained in the samples. Particularly, these indices estimated the abundance of the community. The algorithms for the two differed, with larger Chao and ACE indices indicating a greater abundance of species in the sample communities. The ACE index and Chao index of the depression group community were both significantly lower than those of the healthy comparison group (*p* < .05), as seen in Figures 6(c) and 6(d).

Coverage refers to the coverage of each sample library. The higher its value, the lower the probability of microorganisms in the sample whose sequences were not determined, which reflects whether the sequencing results represent the true condition of the sample. In this study, the coverage index of the depression group and the healthy comparison group communities was approximately 0.99842 and 0.99822, respectively. Because the values were both close to 1, it indicates that the sequencing results truly reflected the distribution of microbial populations in the samples.

### 3.6. Gut Microecological Composition and Distribution Abundance in the Depression Group

We investigated the structure of the fecal microbial community of depressed patients by comparative analysis between the sequenced samples and the fecal microbial community of the corresponding healthy individuals. We performed species heat map analysis based on the relative abundance of each species in each sample and log-transformed the relative abundance to a base of 10, since the relative abundance of species can vary widely and affect sample clustering. The fecal flora sequences of the depressed and healthy control populations belonged mainly to four phyla, including the phyla Thick Bacterial Wall, Bacteroides, Actinobacteria, and Aspergillus, with the vast majority belonging to the Thick Bacterial Wall and Bacteroides phyla, which are the dominant bacteria in the intestinal flora. The differences in microbial community abundance between the samples of the two groups were examined statistically, and the significance of the differences was assessed using the FDR.

At the phylum classification level, both the depressed and healthy comparison groups had the highest abundance of Firmicutes, followed by Actinobacteria, and there was no significant difference between the two groups at this level (*p* < .05, FDR > 0.1). At the phylum classification level, both the depressed and healthy comparison groups had the highest abundance of Clostridia, and there was no significant difference between the two groups at this level (*p* < .05, FDR > 0.1). At the level of order classification, Clostridiales was the most abundant in both the depressed and healthy comparison groups, and there was no significant difference between the two groups at this level (*p* < .05, FDR > 0.1) At the family level, the depressed group had the highest abundance of Lachnospiraceae, while the healthy comparison group had the highest abundance of Ruminococcaceae, but there was no significant difference between the two groups at the level of both Lachnospiraceae and Ruminococcaceae (*p* < .05, FDR > .1). At the genus level, the depressed group had the highest abundance of Bifidobacterium, and the healthy comparison group had the highest abundance of Faecalibacterium, but there was no significant difference between the two groups at the level of both Bifidobacterium and Faecalibacterium (*p* < .05, FDR > 0.1). At the species level, compared to the healthy comparison group, the depression group had the highest abundance of *Coprococcus catus* (0.006762 vs. 0.038359, *p* < .05, FDR < .1), while the relative abundance of *Bacteroides barnesiae* (0.000047 vs. 0.092532, *p* < .05, FDR < .1) was significantly reduced compared to the healthy comparisons. The mean abundances of samples from both groups at the species level are shown in Table 5.

## 4. Discussion

Depression is a common affective disorder with a high incidence and lethality, which seriously affects the health and quality of life of patients and places a great burden on their families and society [28]. Previous studies on the pathogenesis of depression focused on neurotransmitter defects [29], neurotrophic alterations [30], and endocrine system dysfunction [31]; however, increasing attention is being paid to the role of environmental factors and immune dysregulation in the pathogenesis of depression. As the metagenomic study of the human gut microbial community continues to progress, novel molecular biological evidence has revealed that the balance and function of the species, composition, and quantity of the gut microbial community not only participate in the regulation of physiological functions of the body but also new evidence shows that they can participate in the regulation of higher neurological activities through the brain gut axis [32–34]. The “brain-gut axis” regulation is closely related to psychosomatic health and diseases (e.g., anxiety, depression, cognitive impairment, schizophrenia, and Alzheimer's disease) [35].

The brain-gut axis is a bidirectional regulatory axis between the gastrointestinal tract and the brain, including the enteric nervous system (ENS), central nervous system (CNS), autonomic nervous system (ANS), and the HPA axis [35]. The gastrointestinal tract has motor and sensory functions and is the only organ in the body that is jointly governed by the ANS, ENS, and CNS. It is widely known as the “emotional reactor.” If the gastrointestinal tract is uncomfortable, it can trigger an emotional response, activating neural activity in the CNS. This neural activity transmits regulatory information to the gastrointestinal tract via the gut-brain axis, causing changes in its secretory function and dynamics, activating intestinal mucosal immunity, and affecting the mucosal barrier function of the intestine [36]. This suggests that the brain-gut axis may play an important role in the development of psychiatric disorders. The interaction of microorganisms colonizing the gut allows them to participate in the function of the brain-gut axis. In other words, there is a bidirectional regulation between the gut flora and the brain, such that an imbalance in the gut flora may affect the behavior, mood, and neurotransmitter expression of the host patient through the regulation of immune function [37, 38]. In this study, we attempted to investigate the species diversity and abundance of intestinal microecosystems in depressed patients as a first step in exploring the relationship between depression and intestinal flora, aiming to provide data on the etiology of depression and improve its prevention and treatment methods.

By analyzing the sequencing data of stool samples from patients with depression and healthy comparisons, we found that gut flora diversity was significantly lower in the depressed group than in the healthy comparisons. It is now generally accepted that decreased intestinal flora diversity is detrimental to human health and is commonly associated with obesity, inflammatory bowel disease, and antibiotic administration [39–41]. In particular, it has been reported in the literature that intestinal flora diversity is significantly reduced in patients with inflammatory bowel disease [40] and gradually rebounds as the disease recovers. However, the role of gut flora diversity in depression remains controversial. Kelly et al. [42] showed that depression is associated with alterations in the composition of the gut microbiota, usually in the form of reduced abundance and diversity, by studying the gut flora of 34 depressed patients, which is consistent with the results of the present study. Naseribafrouei et al. [43] observed the gut microbial structure in patients with depression, but found no significant difference in gut flora diversity from that of healthy comparisons, which is inconsistent with the results of our study. The results reported by Naseribafrouei et al. may be influenced by the fact that the control group comprised outpatients in neurology. Although the disease was not finally diagnosed, their control group may have been under some psychological stress. However, the patients that comprised the control group in our study were deemed healthy and free from psychological and psychiatric disorders.

To demonstrate the effect of depressed mental states on the gut microbiome, one study used an animal model to establish a cause-and-effect relationship between the two and found that the relationship between depressed mental states and the gut microbiome in humans was quantitatively different than in mice [44]. However, it was not possible to determine whether the psychological state of depression is a cause or an effect of the changes in gut microbiota diversity. Understanding the causal relationship between the two would shed light on the role of the gut microbiota in depression. This can be inferred from the chronology of depression and changes in the gut flora. There are three possible chain reactions between the gut microbiota and depression. First, reductions in species-specific gut flora populations may precede reductions in neurotransmitter levels in the brain, leading to depression. Second, depressive states may lead to alterations in specific gut flora, ultimately leading to more severe depression. Third, because the gut microbiota interacts with the brain via neuroimmune, neuroendocrine, and neural pathways, changes in the entire gut microbiota are relevant to the blood state.

In the present study, the relative abundance of *Coprococcus catus* and *Bacillus pseudomallei* in the stool of the patients in the depression group was significantly lower than that in the control group. *Coprococcus catus* belongs to the thick-walled phylum. Kasai et al. [45] observed that the abundance of *Coprococcus catus* is closely associated with obesity and can be involved in the metabolic process of converting polysaccharides into short-chain fatty acids (SCFAs). A decrease in *Coprococcus catus* abundance tends to cause a decrease in SCFAs. SCFAs are not only an important source of energy for intestinal epithelial cells, but they also affect the intestinal mucosal barrier, permeability of intestinal epithelial cells, oxidative stress, and more. Therefore, we hypothesized that the reduced abundance of *Coprococcus catus* in the intestine may be associated with increased intestinal mucosal permeability in patients with depression. In addition, SCFAs can also promote 5-hydroxytryptamine (5-HT) secretion, enhance colonic contraction, and accelerate transmission; therefore, we hypothesized that a reduced abundance of *Coprococcus catus* may also be associated with impaired gastro-dynamics in patients with depression. In conjunction with another study, it was found that the development of depression is associated with the dysregulation of central emotional neurotransmitters. For instance, low concentrations of “happy” substances, such as 5-HT, dopamine, and endorphins, as well as high concentrations of “unpleasant” molecules, may be associated with depression. It has been found that 5-HT is produced by intestinal chromophores in the gastrointestinal tract [46]. In summary, we hypothesize that the decrease in SCFAs is caused by a decrease in *Coprococcus catus* abundance, causing a decrease in 5-HT secretion and a subsequent increase in intestinal mucosa permeability, gastric motility disorder, and depressed mood.

We also found that the abundance of *Bacteroides barnesiae* belonging to the Anaplasma genus was significantly reduced in patients with depression. The Anaplasma genus is one of the most abundant gram-negative genera in the human gut, accounting for 25% of the total intestinal microbiota [47]. Otaru et al. [48] demonstrated that 90% of the Anaplasma genome (96% in human intestinal isolates alone) contains all the genes required for the production of GABA, suggesting that the genus Anaplasma plays an important role in the regulation of the GABA system in the human gut. There is growing evidence that gut microbes also produce metabolites (neurotransmitters) with high neuroactive potential, including norepinephrine, tryptamine, serotonin, dopamine, and GABA [49, 50]. In turn, these microbiota-derived neurotransmitters can regulate host homeostasis within the gastrointestinal tract, at distant body sites (e.g., the brain), and in complex neuronal, immune, and humoral signaling cascades (i.e., the gut-brain axis) [51, 52]. Furthermore, there is other evidence that bacteria-derived GABA may be a key neuroimmune modulator, linking the gut microbiota and mental health [24]. The exact functions and benefits of these neurotransmitters produced by gut microbes, the mechanisms regulating their production in the gut ecosystem, and their interactions with the gut and peripheral tissues remain largely unexplored. In summary, we speculate that *Bacteroides barnesiae* may modulate human mental health through the production of GABA and thus act as a key neuroimmune modulator.

In conclusion, we found the relative abundance of *Coprococcus catus*, *Bacillus pseudomallei*, and *Bacteroides barnesiae* belonging to the Anaplasma genus in the stool of the patients in the depression group was significantly lower than that in the control group. Valles-Colomer et al. [50] compared the fecal microbiota composition in patients with major depressive disorder (MDD) and healthy individuals. Reduced levels of Faecalibacterium, an important butyrate producer, were observed in patients with MDD. Davey et al. [53] found that *Coprococcus* spp. were also depleted in depression. Here, we suspect different findings around abundance of species; genus may refer to the same microbial metabolites involved in the pathophysiology of major depressive disorder.

Although alterations in bacterial abundance were observed in this study, it is important to recognize that there was atypical antipsychotic use in a subset of the included patients in the depression group. Atypical antipsychotic use often results in increased body weight, and alterations in body weight and gut flora are closely related. Davey et al. found that olanzapine not only had some antibacterial activity against intestinal colonizing bacteria but also increased the abundance of the thick-walled phylum and decreased the abundance of the anaphylum in the rat intestine in vitro. This alteration trend was similar to the gut flora in the obese population [54, 55]. Although strict inclusion criteria were set for this study to control for potential confounders, we were unable to completely exclude the effect of atypical antipsychotic use. This is one of the most significant limitations of this study; therefore, future studies should include first-episode patients to minimize the effects of atypical antipsychotic use.

In addition, there were other limitations to this study. First, this was a cross-sectional study that could only demonstrate that the gut flora of depressed patients differed from that of healthy individuals. Second, the bacteria corresponding to the important OTUs screened were not validated, and since they could neither be cultured nor purchased commercially, their interactions with the host were not studied.

## 5. Conclusions

In conclusion, our findings demonstrate that depression is closely related to the intestinal microecological system and that the intestinal microecological system may influence the development of depression either through an indirect mode of microbial metabolism or through direct activation, such as the activation of the immune system. Our comprehensive study of the structure of depression-related microecological systems enriches the etiological theory of depression and lays the foundation for the application of microecology-related therapeutic approaches in preventing and treating depression.

## Figures and Tables

**Figure 1:** Flowchart showing the total number of participants enrolled and the final number of participants included in the study. Forty with depression and 22 healthy comparisons were enrolled in the study.

**Figure 2:** Figure showing the results of OTU Venn diagram. Different color graphics in the diagram represent different groups. The number of overlapping parts between different color graphics is the number of OTUs shared between the two samples or two groups. OTU Venn diagrams yielded 356 OTUs in the depression group and 248 OTUs in the healthy comparison group, for a total of 800 OTUs in both groups.

**Figure 3:** Principal component analysis of depression and healthy comparison groups. The relative abundance of each OTU in each sample can be calculated according to the abundance file of OTU in each sample; this abundance information can be used for PCA analysis of OTU and to analyze statistics and mapping through Ade4 package in R (v3.1.1) language. The abscissa represents the first principal component, the ordinate represents the second principal component, and the percentage in brackets represents the contribution value of the first and the second principal components to the sample difference, respectively. The midpoint of the figure represents each sample, respectively, and different colors represent that the samples belong to different groups.

**Figure 4:** The species profiling of each sample at different classification levels. By comparing with the database, OTU species are classified, and the area map and histogram of each sample species are, respectively, profiled at the classification levels of phylum, class, order, family, genus, and species. From the figure, we can intuitively see the proportion of different species in each sample. (a) The species profiling of each sample at phylum level. (b) The species profiling of each sample at class level. (c) The species profiling of each sample at order level. (d) The species profiling of each sample at family level. (e) The species profiling of each sample at genus level. (f) The species profiling of each sample at species level.

**Figure 5:** Rank abundance curve of bacterial OTUs derived from two groups. The Rarefaction curves use the relative proportion of various OTUs known in the measured sequence to calculate the expected value of each alpha index when *n* tags (*n* is less than the total number of measured reads sequences) are extracted and then draw the curve according to the expected value of a group of *n* values (generally a group of equal difference series less than the total number of sequences, and the common deviation of this project is 500) and their corresponding alpha index.

**Figure 6:** Box diagram of alpha diversity between groups, which more intuitively shows the differences of alpha diversity between groups. The box chart can display 5 statistics (minimum, first quartile, median, third median and maximum, and 5 lines from bottom to top), and the outliers are marked with “0”.

**Table 1:** 16S rDNA V3-V4 region amplification reaction system.

Ingredients	Volume (*μ*L)
Q5 high-fidelity DNA polymerase	0.25
5∗ reaction buffer	5
5∗ high GC buffer	5
dNTP (10 mM)	2
Template DNA	2
Forward primers (10 *μ*M)	1
Reverse primer (10 *μ*M)	1
Water	8.75

**Table 2:** Descriptive characteristics of subjects with depression and healthy comparison group.

Characteristics	Depression	Healthy comparisons	*p* value^1^
Number	40	22	-^2^
Age (mean ± SD years)	37.9 ± 14.3	44.0 ± 14.3	.803
Sex {M, *n* (%)}	15 (37.5)	13 (59.1)	.118
Alcohol intake {yes, *n* (%)}	14 (35.0)	13 (59.1)	.108
Smoking {yes, *n* (%)}	15 (37.5)	12 (54.5)	.285
Laboratory data	Depression	Healthy comparisons	*p* value^1^
Total cholesterol (mean ± SD mmol/L)	4.4 ± 0.8	5.3 ± 1.0	.185
Triglyceride (mean ± SD mmol/L)	1.7 ± 0.7	1.9 ± 0.8	.990
Glucose (mean ± SD mmol/L)	4.5 ± 0.5	5.0 ± 0.6	.074
AST (mean ± SD U/L)	20.3 ± 7.3	25.7 ± 7.1	.676
ALT (mean ± SD U/L)	20.1 ± 9.7	17.4 ± 8.7	.184

Abbreviation: ALT: alanine aminotransferase; AST: aspartate aminotransferase. ^1^*p* values are based on two-sample *t*-test for continuous variables and Fisher's exact test for categorical variables. ^2^No comparison between two groups.

**Table 3:** OTU number of samples with depression and healthy comparison group.

Sample name	Tag number^1^	OTU number	Sample name	Tag number	OTU number
C01	41329	249	C02	44779	206
C03	42667	264	C04	43422	205
C05	42219	155	C06	35181	179
C07	41529	207	C08	22876	349
C09	42642	229	C10	50882	346
C11	41526	299	C12	40933	319
C13	35381	360	C14	35524	377
C15	38949	351	C16	40531	257
C17	40633	239	C18	41118	207
C19	42872	190	C20	33470	423
C21	36544	298	C22	38323	360
M01	37116	194	M02	40851	129
M03	34214	215	M04	31553	209
M05	47396	169	M06	34412	299
M07	40783	181	M08	48143	138
M09	42329	224	M10	40270	195
M11	37059	292	M12	49738	306
M13	43366	203	M14	31752	234
M15	48224	207	M16	44172	159
M17	44842	192	M18	38513	248
M19	36113	204	M20	50219	231
M21	33372	251	M22	44141	136
M23	41347	241	M24	36027	201
M25	18809	422	M26	40426	237
M27	46523	364	M28	43689	199
M29	48436	174	M30	41852	202
M31	44213	154	M32	43299	177
M33	41459	190	M34	36706	252
M35	32653	290	M36	36821	270
M37	44723	196	M38	39866	248
M39	48049	186	M40	53369	293

^1^Tag number: the total number of tags in the sample that can be aligned with OTU representative sequences and OTU has annotation results.

**Table 4:** Sequencing results and flora diversity index of samples from depression and healthy comparison group.

Group	OTU number^1^	Shanno^2^	Simpson^2^	ACE^2^	Chao 1^2^	Coverage^2^
MDD	356	2.21889 ± 0.55610	0.26652 ± 0.13106	310.58598 ± 64.37160	292.43980 ± 58.23966	0.99842 ± 0.00059
HCs	248	2.73621 ± 0.49996	0.16903 ± 0.07355	361.12332 ± 68.02326	346.52272 ± 70.84198	0.99822 ± 0.00048
*p* value^3^	-^4^	.00096	.00207	.00385	.00331	.03290

^1^The operational taxonomic units (OTUs) were defined with 97% similarity level. ^2^The coverage percentage, the richness estimators (ACE and Chao1), and diversity indices (Shannon and Simpson) were calculated using the Mothur program (v1.31.2), respectively. The data are expressed as mean + SD. ^3^*p* values are based on Wilcoxon Rank-Sum test. ^4^No comparison between two groups.

**Table 5:** Comparison of microbial community abundance between depression and healthy comparison group.

Species	HCs		MDD		*p* value^1^	FDR^2^
	Mean	SD	Mean	SD		
*Coprococcus catus*	0.038359	0.058721	0.006762	0.012516	.000331	0.028135
*Bacteroides barnesiae*	0.092532	0.42721	4.70E-05	0.000296	.002833	0.080268
*Butyricicoccus pullicaecorum*	0.375932	0.599498	0.080343	0.13615	.004823	0.102408
*Plesiomonas shigelloides*	0.001833	0.004804	0	0	.006024	0.102408
*Parabacteroides distasonis*	0.151698	0.391676	0.021075	0.038717	.009905	0.140321
*Bifidobacterium longum*	1.693232	4.071802	4.246913	8.39315	.017499	0.19244
*Prevotella copri*	5.208903	14.272321	1.000945	4.521655	.018112	0.19244
*Bacteroides uniformis*	0.500099	0.687801	1.009413	4.695555	.022927	0.216533
*Akkermansia muciniphila*	0.03665	0.080272	0.196297	1.172834	0.034624	0.294304

^1^The Metastats software was used to analyze the significant differences between groups. The *p* value is corrected by *p*.adjust in the R package. The correction method is Benjamini-Hochberg (BH). ^2^False discovery rate (FDR) was used to assess the significance of the difference.

## Data Availability

The datasets analyzed during the current study are available from the corresponding author on reasonable request.

## Abbreviations

HPA: Hypothalamic pituitary adrenal
NMDAR: N-methyl-D-aspartate receptor
GABA: Gamma-aminobutyric acid
MGBA: Microbiota-gut-brain axis
ICD-10: International Statistical Classification of Diseases and Related Health Problems 10th Revision
PCR: Polymerase chain reaction
QC: Quality control
FLASH: The Fast Length Adjustment of Short reads
OTU: Operational taxonomic unit
PCA: Principal component analysis
FDR: False discovery rate
BH: Benjamini-Hochberg
ALT: Alanine aminotransferase
AST: Aspartate aminotransferase
ENS: Enteric nervous system
CNS: Central nervous system
ANS: Autonomic nervous system
SCFAs: Short-chain fatty acids
5-HT: 5-Hydroxytryptamine.
